# IoMT Meets Machine Learning: From Edge to Cloud Chronic Diseases Diagnosis System

**DOI:** 10.1155/2023/9995292

**Published:** 2023-06-01

**Authors:** Natasha Nigar, Abdul Jaleel, Shahid Islam, Muhammad Kashif Shahzad, Emmanuel Ampoma Affum

**Affiliations:** ^1^Department of Computer Science (RCET), University of Engineering and Technology, Lahore, Pakistan; ^2^Power Information Technology Company (PITC), Ministry of Energy,Power Division, Government of Pakistan, Lahore, Pakistan; ^3^Department of Telecommunication Engineering, Kwame Nkrumah University of Science and Technology, Kumasi, Ghana

## Abstract

In conventional healthcare, real-time monitoring of patient records and information mining for timely diagnosis of chronic diseases under certain health conditions is a crucial process. Chronic diseases, if not diagnosed in time, may result in patients' death. In modern medical and healthcare systems, Internet of Things (IoT) driven ecosystems use autonomous sensors to sense and track patients' medical conditions and suggest appropriate actions. In this paper, a novel IoT and machine learning (ML)-based hybrid approach is proposed that considers multiple perspectives for early detection and monitoring of 6 different chronic diseases such as COVID-19, pneumonia, diabetes, heart disease, brain tumor, and Alzheimer's. The results from multiple ML models are compared for accuracy, precision, recall, F1 score, and area under the curve (AUC) as a performance measure. The proposed approach is validated in the cloud-based environment using benchmark and real-world datasets. The statistical analyses on the datasets using ANOVA tests show that the accuracy results of different classifiers are significantly different. This will help the healthcare sector and doctors in the early diagnosis of chronic diseases.

## 1. Introduction

Healthcare has an undeniable impact on the well-being of individuals [1, 2]. Chronic diseases adversely affect the health of human beings. This requires an early and accurate diagnosis which is possible after a physical examination in the hospital. The delayed diagnosis requires patients' admission to the hospital for treatment which results in increased healthcare cost and duration, and restricted healthcare facilities in rural and remote areas [3]. The traditional diagnosis approaches are human-centered and error-prone, e.g., missed or delayed diagnosis, failure to initiate the follow-up, inaccessible patients' history, wrong medical prescription, and incomplete information about patient history which may lead to severe consequences to patients' health [4]. These challenges require the healthcare domain to adopt the latest technological disruptions in the fields of IoT, artificial intelligence (AI), and ML to reduce human error.

The IoT has demonstrated its benefits in connecting medical devices, sensors, and healthcare professionals to provide quality medical services [5] which resulted in extended healthcare services and reduced costs. The medical history of patients collected through these IoT devices also helps in the effective monitoring of patients' health and early diagnosis by healthcare service providers. These benefits have resulted in the transformation of present healthcare facilities from hospital-centric facilities to patient-centric facilities [6, 7]. The network of medical devices and healthcare professionals created through sensors is also referred to as the Internet of Medical Things (IoMT) which in a healthcare system is called healthcare Internet of Things (HIoT) [8].

The IoMT has revolutionized the healthcare industry and demonstrates effective healthcare and monitoring system. This connects device to machine, doctor to doctor, patient to doctor, object to object, patient to machine, doctor to machine, sensors *o* mobile, and mobile to human in an intelligent way [4]. The effective usage of IoT devices data is critical and key to success. In this context, ML has proved to be one of the most suitable computational paradigm which offers embedded intelligence in the IoT devices [9] for predictive and prescriptive diagnosis in healthcare.

The existing systems are mostly limited to the prediction of one chronic disease considering no computing layer. To overcome such issues, an ML-based predictive model is presented to improve the diagnosis of six different chronic diseases based on the conceptual framework of 3 different computing layers, i.e., edge computing, fog computing, and cloud computing. The IoT devices (smart devices) data are used for diagnosis using 3 different computing techniques with the following contributions:

- New system design: a novel system architecture is designed using IoMT and ML, based on a conceptual framework of 3 different computing layers, for accurate and quick diagnosis of 6 different chronic diseases
- State-of-the-art algorithms comparative study: different ML-based states of the art algorithms are compared for chronic diseases diagnosis
- Data set: the proposed approach is tested on both real-world and benchmark data instances from Kaggle [10]

This paper is structured into six sections.  Section 2 presents the background and related work whereas the proposed methodology is explained in Section 3. The experimental design and analysis results are presented in Section 4. The threats and validity of this study are presented in Section 5. The paper concludes with Section 6 where results and future directions are presented.

## 2. Literature Review

### 2.1. Background

The healthcare industry is rapidly adopting the IoT by integrating technology into medical devices to enhance the quality and efficiency of service [11]. On the other hand, the advancement in machine learning has influenced researchers to predict chronic diseases with high accuracy. This ML-based IoMT framework is playing a significant role in the healthcare industry by reducing the mortality rate by the early detection of diseases [12]. Existing studies analyze mostly one chronic disease [11, 13–17]. However, there are many other chronic diseases exist, e.g., pneumonia, COVID-19. In this regard, we investigate the performance of state-of-the-art algorithms to diagnose chronic diseases. The reason for selecting these algorithms is that they are simple to implement and most of them are open source.

The convolution neural network (CNN) [18] is a dominant ML approach for image recognition, image classification, and object detection. It is a high-performance classifier that automatically detects the important features and is computationally efficient. The basic structure of CNN is given in Figure 1. The VGG16 [19] is based on a CNN architecture that is used for object detection and classification. It utilizes 16 layers with weights and is considered one of the best image classification algorithms. However, it is very slow to train. The VGG19 [19] is also a CNN that is based on 19 deep layers. The first 16 convolutional layers are used for feature extraction, and the rest 3 layers for classification. It is trained on more than a million images from the ImageNet database and can classify images into 1000 object categories. It is a very popular method due to the use of multiple 3 × 3 filters in each convolutional layer.

Residual network (ResNet) [20] is one of the most powerful deep neural networks which have achieved excellent performance to solve classification problems. It is based on CNN architecture to support hundreds or thousands of convolutional layers. DenseNet [21] is also a CNN-based architecture that utilizes dense connections among layers through dense blocks. It makes direct connections between any two layers with the same feature-map size. It has proved to yield consistent improvement in accuracy without any signs of performance degradation or overfitting. The Inception-v3 [22] is a pretrained model on the ImageNet datasets. It performs better for image classification problems as compared to other deep learning algorithms. XGBoost [23] is a decision tree-based ML algorithm that combines the results of many models, called base learners to make a prediction. It is a sequential model where each subsequent tree is dependent on the outcome of the last. It is a highly flexible technique and handles missing values automatically.

Decision tree (DT) [24] is a most popular nonparametric supervised learning algorithm that is used for classification and prediction. They support scalability for large datasets, handle imbalanced datasets, and easy to use. However, they can be computationally expensive to train and suffer from high variance. To overcome the issue of high variance, we apply bagging. In bagging, bootstrap samples are created from the training data set, and then, trees are built on bootstrap samples. After that, the output is aggregated from all the trees to predict the final output [25]. Random forest (RF) [26] is a widely used ML algorithm due to its ease of use and flexibility. It handles both classification and regression problems and combines the output of multiple decision trees to reach a single result. It also offers feature selection to quickly understand the important or nonimportant features that are affecting the final result.

### 2.2. Related Works

Wearable/smart IoT devices are used in healthcare for real-time monitoring of patients' health. The ML models developed based on the data collected from these IoT devices have been successful in accurately diagnosing the diseases. In this section, a literature review of recent IoT-driven ML model-based approaches is presented.

Khelili et al. [27] proposed an IoMT CNN-based model to detect COVID-19 cases from pneumonia and normal cases with 97% accuracy. Rani et al. [28] presented an IoMT with ML-based COVID-19 diagnosis model. They used AdaBoost with random forest (AB-RF), artificial neural network (ANN), support vector machine (SVM), and DT as classifiers. Parthasarathy and Vivekanandan [14] developed a diagnosis model for arthritis disease. In this model, data were collected from sensors and stored on cloud whereas an optimization algorithm considers swelling and uric acid as key predictors. Bhuvaneswari and Manikandan [15] proposed a novel framework based on ML for type-2 diabetes analysis.

Rohani et al. [29] developed a brain-computer interface (BCI) system for the rehabilitation of attention deficit hyperactive disorder in children. They applied SVM [30] using temporal and template-based features for disorder diagnosis. Monteiro et al. [31] proposed a system based on ML techniques to predict Ischemic stroke. Palani and Venkatalakshmi [32] proposed an IoT-based predictive model using fuzzy cluster to predict lung cancer through continuous monitoring. The proposed system also improved healthcare delivery through real-time medical instructions. Sciarrone [33] developed a reliable wearable and noninvasive device to detect Alzheimer's and Parkinson's disease.

Kumar and Devi Gandhi [13] presented an IoT architecture employing ML algorithms for the early detection of heart diseases. The proposed architecture comprises data collected from wearable smart devices with storage on the cloud and prediction using the regression-based local model. Alamelu and Thilagamani [16] developed a lion-based butterfly optimization algorithm with an improved YOLO-4 model to predict heart disease. Prakash and Karthikeyan [17] also proposed a dual-layer deep ensembling technique to classify the heart disease by outperforming traditional state-of-the-art classifiers. Khan [11] presented a modified deep convolutional neural network to diagnose the heart disease. As an improvement of their work [12] to predict the heart disease, they also proposed an optimized algorithm in an IoMT cloud environment.

Ogundokun et al. [34] proposed an hybrid technique based on Inception-v3 and SVM to detect the human posture in health monitoring systems. The same effort [35] has been made to identify the human activity using the IoMT approach to avoid fall detection, smoking control, sportive exercises, and monitoring of daily life activities. Ogundokun et al. [36] developed a hyperparameter-optimized neural network technique to diagnose the breast cancer.

Kim and Chung [37] proposed a model to keep track of chronic diseases as full recovery from such diseases is rare due to diverse causes and complexity. Farahani et al. [38] presented a comprehensive survey based on the multilayer architecture of IoT e-health that includes devices, fog, and cloud computing to enable the system to support latency, variety, and speed of data processing. Moreover, challenges such as scalability, data management, interoperability, privacy, and security are also considered for complex data processing in the IoT *e*-health environment. Pal et al. [39] proposed a novel method for real-time detection of anomalies in the patients' data. The studies [40, 41] proposed a secure framework to ensure the privacy of patients' data. Besides these, other studies [8, 42–44] provide a survey of research on the IoT in healthcare. All of these studies have also been summarized in Table 1.

The above literature highlights that most of the studies focus on a single disease using cloud excluding many chronic diseases and computing layers. Human life is afflicted by various diseases; therefore, this raises interest in research to consider chronic diseases.

## 3. Proposed Methodology

In this section, the proposed methodology for six chronic diseases is presented followed by the ML model (Figure 2) and three different computing layers to detect these diseases.

The proposed methodology is divided into three modules:

- Data fetching
- Disease detection
- Computing layers

### 3.1. Data Fetching

In this module, data are fetched from different smart or wearable IoT devices, e.g., cameras and smart watches. Consequently, data are fed into the system.

### 3.2. Disease Detection

This module is focused on developing the ML model. The fetched data from the previous module are processed using different state-of-the-art ML algorithms for multichronic disease diagnosis. The ML model uses images to diagnose COVID-19, brain tumor, pneumonia, and Alzheimer. The workflow of the proposed methodology is presented in Figure 3. The detailed steps for this process are explained as follows:

- Data preprocessing: In this step, images are cropped and resized to obtain the region of interest (ROI). This step increases the performance and reliability of the trained classifier and reduces the respective computation time.
- Data augmentation: In image classification, data augmentation is a technique to flip, rotate, and crop the image. Due to the limited availability of the dataset, this technique is applied to available images to maximize the effective usage of our limited training samples and to improve the model's accuracy.
- Feature extraction: The default feature extraction technique is applied to generate multiple features to improve disease detection.

For heart disease, both numerical and categorical values are input to the classifier. First, the dataset is divided into training and test datasets in 70% and 30% ratio, respectively. Subsequently, a categorical feature encoding technique is applied to convert categorical values into integer format to improve the ML model's learning efficiency. The Bayesian optimization [54] is applied for hyperparameter optimization because all prediction systems with efficient hyperparameter tuning achieve better results [55]. The XGBoost algorithm [48] is used to train the model. It is a tree-based distributed ML classification algorithm used to improve the model's speed and performance up to 10 times in comparison to other classification algorithms [55]. In each iteration, Bayesian optimization tries to improve the AUC mean score. The workflow of this proposed methodology is presented in Figure 4.

In case of diabetics' disease diagnosis, the input to the system is in the form of numerical values. The first step is to standardize the data due to varying scale and division in 70% and 30% ratio as training and test dataset. The visual representation of the proposed methodology is also shown in Figure 5.

### 3.3. Computing Layers

The computing module comprises of 3 layers architecture to deploy the ML algorithm on a server depending on the patient's crowd. We consider that if the number of patients is limited, our model is embedded in the Arduino module; otherwise, if the patients' count exceeds a certain threshold, we use edge computing for training our model. Moreover, for a huge count of patients, the classifier is placed in the cloud server.

## 4. Experimental Analysis

### 4.1. Experimental Setup

#### 4.1.1. Dataset

In this paper, six datasets for six different chronic diseases are used (Table 2). For COVID-19, diabetes, and heart diseases, the real-time dataset is used. However, to diagnose the brain tumor and pneumonia, the dataset is obtained both from Kaggle [10] and real data. The open access series of imaging studies (OASIS) [56] and real datasets are used for Alzheimer's disease.

#### 4.1.2. Performance Measures

In this section, the quantitative metrics used to evaluate the performance of classifiers are presented. As results are classified as a positive class or negative class in the classification problems, therefore, there are four possible states also known as confusion matrix [59].

- True positive (TP): accurate classification of positive class
- True negative (TN): accurate classification of negative class
- False positive (FP): inaccurate classification of positive class
- False negative (FN): inaccurate classification of negative class

The results' performance is evaluated using accuracy, precision, recall, and F1 score, which are calculated as follows:

(1) $$\begin{array}{c} Accuracy=\frac{TP+TN}{FP+TN+TP+FN}\text{,} \end{array}$$

(2) $$\begin{array}{c} Precision=\frac{TP}{TP+FP}\text{,} \end{array}$$

(3) $$\begin{array}{c} \frac{Recall}{Sensivity}=\frac{TP}{TP+FN}\text{,} \end{array}$$

(4) $$\begin{array}{c} Specificity=\frac{TN}{TN+FP}\text{,} \end{array}$$

(5) $$\begin{array}{c} F1=2.\frac{precision.recall}{precision+recall}\text{.} \end{array}$$

The AUC is also used as a performance metric. It is measured by plotting a ROC (receiver operating characteristic) curve of the true positive rate against the false positive rate at different classification thresholds. The term “AUC = 1” indicates that the classifier is able to perfectly distinguish between all the positive and the negative classes correctly. If, however, the AUC is 0, then the classifier is predicting all negatives as positives, and vice versa.

- True positive rate (TPR): it is also known as recall or sensitivity as defined in (3)
- False positive rate (FNR) = (*FP*)/(*FP*+*TN*) = (1 − specificity (4))

#### 4.1.3. Parameter Settings

In Table 3, the hyperparameter settings used for COVID-19, pneumonia, brain tumor, and Alzheimer's diseases are presented whereas Table 4 presents the hyperparameter settings for heart disease diagnosis.

#### 4.1.4. Experimental Environment

All the experiments are run on GPU-enabled TensorFlow [60] with Keras [61] framework using Python programming language, running on a personal computer with Intel core i5, 3.2 GHz CPU, and 16 GB RAM.

### 4.2. Results and Discussion

#### 4.2.1. Comparison of State-of-the-Art Methods

In the proposed methodology, five pretrained deep CNN models, VGG16, VGG19, ResNet, DenseNet, and Inception-v3, are used to detect COVID-19. The results as presented in Table 5 show that the pretrained VGG16 model significantly outperforms the other four models with the highest classification performance as 80%. After the VGG16 classifier, VGG19, DenseNet, and Inception-v3 resulted in an accuracy rate of 60%, whereas ResNet showed the lowest accuracy rate as 50%. The visual representation of these values is also given in Figure 6.

The comparative analysis of four transfer learning models to detect pneumonia using chest X-ray images is presented in Table 6. The results show that VGG19 outperforms its peers as it achieves the highest values for classification accuracy and F1 score as 88.46% and 91%, respectively. However, its recall is less than VGG16. The ResNet and Inception-v3 are the least performing models in terms of accuracy, recall, and F1 score. The visual representation of these results is presented in Figure 7.  Table 7 presents the accuracy and loss values achieved by each model during training and validation. The results also show that ResNet and Inception-v3 show substantial overfitting as the difference between training and validation accuracy is significantly large. These two models have large validation loss, and their validation or classification accuracy is also low. The graphical representation of model accuracy and model loss of ResNet and Inception-v3 is presented in Figures 8(a) and 8(b), respectively. It is evident that there is variation in training, validation accuracies, and loss as the epochs count increases.

For diabetics diagnosis, decision tree, bagging with a decision tree, random forest, and random forest with feature selection method are used. The results show that the random forest with feature selection method demonstrates the highest accuracy measure of 92.02% (Figure 9) whereas the decision tree performed least with an accuracy rate of 75.2% (Table 8). The accuracy is tested with various numbers of trees until the accuracy becomes stable and received a stable accuracy rate from 40 trees.

For brain tumor diagnosis, CNN is used for faster and efficient processing. CNN has proven to give the better performance than traditional ones [62] with an accuracy rate of 91%. However, to detect the heart disease, the XGBoost classifier is applied with Bayesian optimization. We calculate the AUC to measure the performance of our model which resulted in 0.883 as shown in Figure 10. This shows the optimal performance of the model. The confusion matrix is also shown in Figure 11 which shows that the trained classifier made predictions with high accuracy.

The CNN model is used through 15 epochs for Alzheimer's disease. The results show that we reached a general accuracy of 97%.  Figure 12 presents how the training and validation accuracy converges as the epochs progress. Reasonably, there is a convergence towards a higher level of accuracy, the more epochs the model runs through. It can be observed that as the model reaches 10 epochs, we reach notable diminishing returns.

#### 4.2.2. Statistical Analysis

In this section, we perform the analysis of variance (ANOVA) test to analyze the statistical significance of the ML models. ANOVA is a statistical technique to analyze the differences among group means by comparing the variance among groups relative to variance within groups [17]. The *p* value in ANOVA test should be lower than 0.05 (5%) to reject the null hypothesis (*H*_0_) which assumes in our study that the accuracy results of all classifiers are equal.

Thus, this study simulates the different machine-learning methods on chronic disease datasets. This experiment primarily aims on building several machine learning classifiers on different disease datasets and analyzing the accuracies among those classifiers. The accuracy performance of each classifier is compared statistically to determine that either classifier's accuracy is statistically significant from each other. In this experiment, we perform ANOVA test for COVID-19, pneumonia, and diabetes datasets as shown in Table 9.

## 5. Threats to Validity

This study aims to diagnose chronic diseases in a timely and cost-effective manner. However, there are few limitations to this work. First, the inclusion of more real-world scenarios may improve diagnostic accuracy. Besides the fact that available datasets are limited, the inclusion of more real-world instances will improve the scalability and validation of the proposed approach. This will also add resilience to the proposed methodology by generating identical diagnosis as a medical doctor.

## 6. Conclusion

Internet has a major impact on our lives, spanning from professional life to social relationships. The IoT has added a new dimension to this process by establishing communication among smart objects, leading to the vision of anytime, anywhere, any media, and anything communication. IoMT is a specialized version of IoT, which specifically deals with the healthcare domain and is playing a vital role in the healthcare sector to provide cost-effective solutions in terms of hospital billing and waiting time. In this paper, a new approach is presented to diagnose 6 different chronic diseases, namely, COVID-19, diabetes, pneumonia, Alzheimer, heart disease, and brain tumor, using machine learning classifiers based on 3 computing layers. The proposed approach is evaluated for each disease using different classifiers using both benchmark and real-world datasets. This also provides efficient and effective health services to the patients by disseminating the networked information to machine learning classifiers.

In the future, the proposed approach will be evaluated with more real-world datasets while considering more chronic diseases. Moreover, efforts will be made to develop cross-disciplinary chronic disease prediction models due to common feature sets.

## Figures and Tables

**Figure 1:** Structure of CNN.

**Figure 2:** Abstract-level view of the proposed approach.

**Figure 3:** The workflow of the proposed methodology for the diagnosis of COVID-19, pneumonia, brain tumor, and Alzheimer.

**Figure 4:** The workflow of the proposed methodology for the diagnosis of heart disease.

**Figure 5:** The workflow of the proposed methodology for the diagnosis of diabetes.

**Figure 6:** Different ML methods' performance in terms of accuracy, precision, recall, and F1 score for COVID-19.

**Figure 7:** Different ML method performance in terms of accuracy and recall for pneumonia detection.

**Figure 8:** Accuracy and loss graph for pneumonia detection: (a) ResNet performance and (b) Inception-v3 performance.

**Figure 9:** Comparison of different ML algorithms in terms of accuracy for diabetes detection.

**Figure 10:** The AUC for heart disease detection model.

**Figure 11:** Confusion matrix of heart disease detection model.

**Figure 12:** ML model accuracy over several epochs for Alzheimer's dataset.

**Table 1:** Comparative analysis with state-of-art-work for chronic disease detection.

Study	No. of diseases	Disease name	IoT	Methods used	Evaluation metrics	Computing layer
Khelili et al. [27]	1	COVID-19	Yes	CNN	Accuracy, precision, recall, F1 score, AUC	Fog, cloud
Rani et al. [28]	1	COVID-19	Yes	AB-RF, ANN, DT, SVM	Accuracy, F-score	Cloud
Parthasarathy and Vivekanandan [14]	1	Arthritis	Yes	Proposed time wrapping algorithm	ROC analysis using sensitivity and specificity	Personal server, cloud
Bhuvaneswari and Manikandan [15]	1	Type-2 diabetes	No	Modified ant miner tree [45] and genetic algorithm [46]	Accuracy	No
Rohani et al. [29]	1	Attention deficit hyperactive disorder	No	SVM [30]	An average error <30%	No
Monteiro et al. [31]	1	Ischemic stroke	No	Logistic regression [47], SVM [30], decision tree [24], random forest [26], XGboost [48], Astral [49], Dragon [50], Thrive [51]	AUC	No
Palani and Venkatalakshmi [32]	1	Lung cancer	Yes	Modified decision tree and CNN [18]	Accuracy	No
Sciarrone et al. [33]	2	Alzheimer, Parkinson	Yes	Hardware	Accuracy	No
Kumar and Devi Gandhi [13]	1	Heart	Yes	Logistic regression [47]	ROC analysis using sensitivity and specificity	Personal server, cloud
Alamelu and Thilagamani [16]	1	Heart	Yes	Faster R-CNN [52] + SE-Rest-Net-101, improved YOLO-4 [53]	Accuracy	Cloud
Prakash and Karthikeyan [17]	1	Heart	No	Proposed dual-layer deep ensemble techniques	Accuracy	No
Khan [11]	1	Heart	Yes	Modified deep CNN	Accuracy	Cloud
Khan and Algarni [12]	1	Heart	Yes	Modified salp swarm optimization with an adaptive fuzzy inference system	Accuracy, precision	Cloud
Ogundokun et al. [34]	—	Human poster	No	Inception-v3 + SVM	Accuracy, AUC	No
Ogundokun et al. [36]	1	Breast cancer	Yes	Hyperparameter-optimized neural networks	Accuracy	Cloud
Proposed	6	COVID-19, pneumonia, diabetes, heart disease, brain tumor, Alzheimer	Yes	CNN, VGG16, VGG19, ResNet, Inception-v3, XGBoost, decision tree, random forest	Accuracy, precision, F1 score, recall, AUC	Edge, fog, cloud

**Table 2:** Dataset description.

Disease name	Dataset name	No. of instances	No. of attributes	No. of classes
COVID-19	Real	310	—	2
Diabetes	Real	420	14	2
Heart disease	Real	500	13	2
Brain tumor	Kaggle [57] + real	4,262	—	2
Pneumonia	Kaggle [58] + real	6,360	—	2
Alzheimer	OASIS [56] + real	2,000	—	2

**Table 3:** Hyperparameters for the convolutional neural network (CNN) and its' variants classifiers.

Parameters	Values
Input size	256 ∗ 22
Batch size	32
Error function	Categorical cross entropy
Activation	ReLU
Optimizer	SDGM
Learning rate	0.01
Dropout	0.5
Train/Validation	70%/30%

**Table 4:** Hyperparameters for XGBoost classifier.

Parameters	Values
n_estimators	100
max_depth	5
min_child_weight	1
Gamma	0
Colsample	1
Subsample	1
Train/Validation	70%/30%

**Table 5:** Performance results of pretrained ML models for COVID-19.

Models	Accuracy	Precision	Recall	F1 score
VGG16	**0.80**	0.80	**0.80**	**0.80**
VGG19	0.60	0.50	0.625	0.55
ResNet	0.50	0.0	0.0	0.0
DenseNet	0.60	0.50	0.625	0.55
Inception-v3	0.60	1.0	0.55	0.71

Bold values represent that this model value is highest/better as compared to others.

**Table 6:** ML model performance comparison for pneumonia detection.

Models	Accuracy	Recall	F1 score
VGG-16	87.18	96	90
VGG-19	**88.46**	95	**91**
ResNet	77.56	97	84
Inception-v3	70.99	84	78

Bold values represent that this model value is highest/better as compared to others.

**Table 7:** Accuracy and loss values by ML models during training and validation for pneumonia detection.

Models	Training accuracy	Training loss	Validation accuracy	Validation loss
VGG-16	95.61	12.03	87.17	37.94
VGG-19	92.85	18.01	88.46	34.29
ResNet	94.29	14.32	77.56	68.36
Inception-v3	88.96	28.20	70.99	97.56

**Table 8:** ML models performance comparison for diabetes detection.

Models	Accuracy
Decision tree	75.2
Bagging with decision tree	81.3
Random forest	85.6
Random forest with feature selection	**92.02**

Bold values represent that this model value is highest/better as compared to others.

**Table 9:** ANOVA test on classifiers' accuracy results.

Diseases	*P* value				
	Classifiers				
COVID-19 pneumonia	VGG16	VGG19	ResNet	DenseNet	Inception-v3
	0.0003	0.0001	0.0002	0.0004	0.0009
	0.0004	0.0003	0.0007	—	0.0008

Diabetes	DT	Bagging with DT	RF	RF with feature selection	
	0.0001	0.0001	0.0002	0.0003	

## Data Availability

The data supporting the current study are available from the corresponding author upon request.
